# Cardiac Na_v_1.5 is modulated by ubiquitin protein ligase E3 component n-recognin UBR3 and 6

**DOI:** 10.1111/jcmm.12588

**Published:** 2015-06-07

**Authors:** Chunxia Zhao, Lijie Wang, Xiue Ma, Weidong Zhu, Lei Yao, Yingyu Cui, Yi Liu, Jun Li, Xingqun Liang, Yunfu Sun, Li Li, Yi-Han Chen

**Affiliations:** a Key Laboratory of Arrhythmias of the Ministry of Education of China, East Hospital, Tongji University School of MedicineShanghai, China; b Department of Cardiology, Shanghai East Hospital, Tongji University School of MedicineShanghai, China; c Research Center for Translational Medicine, Tongji University School of MedicineShanghai, China; d Department of Pathology and Pathophysiology, Tongji University School of MedicineShanghai, China; e Institute of Medical Genetics, Tongji UniversityShanghai, China

**Keywords:** Na_v_1.5 channel, UBR, cardiomyocyte, degradation, ubiquitin, proteasome

## Abstract

The voltage-gated Na^+^ channel Na_v_1.5 is essential for action potential (AP) formation and electrophysiological homoeostasis in the heart. The ubiquitin–proteasome system (UPS) is a major degradative system for intracellular proteins including ion channels. The ubiquitin protein ligase E3 component N-recognin (UBR) family is a part of the UPS; however, their roles in regulating cardiac Na_v_1.5 channels remain elusive. Here, we found that all of the UBR members were expressed in cardiomyocytes. Individual knockdown of UBR3 or UBR6, but not of other UBR members, significantly increased Na_v_1.5 protein levels in neonatal rat ventricular myocytes, and this effect was verified in HEK293T cells expressing Na_v_1.5 channels. The UBR3/6-dependent regulation of Na_v_1.5 channels was not transcriptionally mediated, and pharmacological inhibition of protein biosynthesis failed to counteract the increase in Na_v_1.5 protein caused by UBR3/6 reduction, suggesting a degradative modulation of UBR3/6 on Na_v_1.5. Furthermore, the effects of UBR3/6 knockdown on Na_v_1.5 proteins were abolished under the inhibition of proteasome activity, and UBR3/6 knockdown reduced Na_v_1.5 ubiquitylation. The double UBR3–UBR6 knockdown resulted in comparable increases in Na_v_1.5 proteins to that observed for single knockdown of either UBR3 or UBR6. Electrophysiological recordings showed that UBR3/6 reduction-mediated increase in Na_v_1.5 protein enhanced the opening of Na_v_1.5 channels and thereby the amplitude of the AP. Thus, our findings indicate that UBR3/6 regulate cardiomyocyte Na_v_1.5 channel protein levels *via* the ubiquitin–proteasome pathway. It is likely that UBR3/6 have the potential to be a therapeutic target for cardiac arrhythmias.

## Introduction

The Na_v_1.5 channel, which is the cardiac isoform of the voltage-gated Na^+^ channel, is critical for the generation of the cardiac action potential (AP) and the conduction of electrical impulses 1. As a membrane protein, the function of Na_v_1.5 in cell electrical excitability not only depends on its own activation but also on the number of Na^+^ channels in the cardiomyocyte plasma membrane 2,3. Although multiple lines of evidence have documented the molecular mechanisms underlying the Na_v_1.5 channel activation, there is a substantial lack of understanding concerning its degradative regulation.

The rapid internalization and degradation of Na_v_1.5 channels have been reported to be associated with the ubiquitin–proteasome system (UPS) 4,5. The UPS, which consists of ubiquitin (Ub), Ub-activating enzyme (E1), Ub-conjugating enzyme (E2), Ub-protein ligase (E3) and the proteasome, is the major degradation pathway of intracellular proteins including voltage-gated channels 4,6. Ub can bind to Na_v_1.5 *via* the E1–E2–E3 enzyme cascade and post-translationally regulate the expression of Na_v_1.5 channels. This process is also a prerequisite for ion channel protein internalization and degradation 7. Ubiquitylation of plasma membrane proteins generally induce their endocytosis, followed by lysosomal or proteasomal degradation 8,9. As a plasma membrane protein, Na_v_1.5 has been observed to be ubiquitylated by a ubiquitin E3 ligase Nedd4-2, which leads to Na_v_1.5 internalization rather than degradation 1,8,10. It remains unclear whether the UPS is involved in the regulation of Na_v_1.5.

In the UPS system, the E3 protein superfamily is the largest family which consists of more than 500 distinct members 11. Among these members, a subfamily termed Ub-protein ligase E3 component N-recognins (UBRs) shares a conserved zinc finger-like 70-residue domain with mammalian E3s and contains at least seven members (UBR1–UBR7). UBR1, UBR2, UBR4 and UBR5 were captured by N-terminal degradation determinants, whereas UBR3, UBR6 and UBR7 were not 12. These UBRs may be involved in Johanson–Blizzard syndrome 13, the sensory system 14 and neurogenesis 15. In addition, UBR1, UBR2, UBR4 and UBR5 in the N-end rule pathway play an important role in cardiac proliferation and hypertrophy 16, angiogenesis 17 and cardiovascular development 15. However, whether UBRs affect the electrical activity of cardiomyocytes remains unknown.

In the present study, we identified the transcript expression profiles of all of the UBR members present in rat cardiomyocytes. Gene knockdown analysis revealed the distinct regulative effects of UBR3 and UBR6 on Na_v_1.5 channels. Further studies showed that UBR3 and UBR6 mediated Na_v_1.5 degradation through the UPS. The UBR3/6-mediated regulation of Na_v_1.5 could change the opening of Na_v_1.5 channels and thereby the amplitude of the APs.

## Materials and methods

### RNA interference

Rat UBR1–UBR7 and human UBR3 and UBR6 were knocked down by specific small interference RNAs (siRNAs) (Jima, Shanghai, China). The scramble control RNA (Shanghai GenePharma Co., Ltd, Shanghai, China) was set up using the 21-nucleotide RNA oligonucleotide that corresponded to the coding sequence of luciferase. All of the siRNA sequences are listed in Table1. Lipofectamine RNAiMAX Reagent (Invitrogen, Carlsbad, CA, USA) was used to transfect the siRNAs into rat cardiomyocytes or HEK293T cells according to the manufacturer’s protocols. The suppression efficiency of UBR1–UBR7 was determined by immunoblotting.

**Table 1:** The siRNA sequences in this study

Species	Target gene symbol	Sequence (5′–3′)
Rat	UBR1	S-GGCCCGACAUCUUAUUGAATT
		A-UCAAUAAGAUGUCGGGCCTT
	UBR2	S-GCGCCACAGAUGAAAUCAATT
		A-UUGAUUUCAUCUGUGGCGCTT
	UBR3	S-GCGGCACUUUAUAAAUUAUTT
		A-AUAAUUUAUAAAGUGCCGCTT
	UBR4	S-CUCCACCACAGAUGAAGAATT
		A-UUCUUCAUCUGUGGUGGAGTT
	UBR5	S-GGGCCUUAUUCCUAAGUAUTT
		A-AUACUUAGGAAUAAGGCCCTT
	UBR6	S-GUCCAAUCCUUGUACAUUATT
		A-UAAUGUACAAGGAUUGGACTT
	UBR7	S-GACUGAACUUAAGGAUUAUTT
		A-AUAAUCCUUAAGUUCAGUCTT
Homo	UBR3	S-CCGUCUUUGAAAGAUUUAATT
		A-UUAAAUCUUUCAAAGACGGTT
	UBR6	S-GCAGACUGGAGGAAUAUAUTT
		A-AUAUAUUCCUCCAGUCUGCTT
Negative control		S-UUCUCCGAACGUGUCACGUTT
		A-ACGUGACACGUUCGGAGAATT

S: sense; A: antisense.

### Isolation of primary neonatal rat ventricular myocytes

All of the animal experiments were approved by the Animal Experiment Committee of Tongji University School of Medicine and conformed to the Guide for the Care and Use of Laboratory Animals (1996) from the U.S. National Institutes of Health. Neonatal rat ventricular myocytes (NRVM) were isolated from the hearts of 1- to 2-day-old Sprague–Dawley rat pups as previously described 18. In brief, after the hearts of the neonatal rats were excised and washed, the ventricles were minced and incubated in a PBS solution containing trypsin (0.25%), collagenase (0.1%) and DNAase (1%) for 5 min. at 37°C. Next, the isolated cells were transferred into a tube containing DMEM supplemented with 10% foetal bovine serum, 100 U/ml penicillin and 100 mg/ml streptomycin. The same procedure was repeated five times to collect a sufficient number of cells. To wash the impurities, the cell pellet was centrifuged and re-suspended. The isolated cells were then purified by differential adhesion for 2 hrs. Finally, the purity of the cardiomyocytes was approximately 98%, as assessed by myocardial troponin immunofluorescence staining. Unsettled cells were washed after 24 hrs, and the medium was replaced daily.

### Cell culture and transfection

The NRVMs and human embryonic kidney 293T (HEK293T) cells were maintained in DMEM supplemented with 10% foetal calf serum (Gibco, Waltham, MA, USA), 1% penicillin and streptomycin in a humidified incubator at 37°C with 5% CO_2_. All of the cells were cultured to 70–90% confluence before transfection. The NRVMs were transfected using the siRNAs. The siRNA of human UBR3/6 as well as Na^+^ channel plasmids (OriGene, Rockville, MD, USA) were cotransfected into HEK293T cells using Lipofectamine 2000 (Invitrogen) according to the manufacturer’s instructions. Exactly, 0.003% SDS and 2 μmol/l MG132 [*N*-[(phenylmethoxy)carbonyl]-l-leucyl-*N*-[(1S)-1-formyl-3-methylbutyl]-l-leu-cinamide were employed to activate or inhibit the proteasome activity respectively.

### RNA extraction, reverse transcription PCR and quantitative real-time PCR

Total RNA was extracted from neonatal rat myocardium and siRNA-treated cells at 48 hrs using TRIzol reagent (Invitrogen) as previously described 19. Reverse transcription PCR (RT-PCR) was conducted using the 1st Strand cDNA Synthesis Kit (TAKARA, Dalian, China) following procedures outlined in the manufacturer’s instructions. Real-time PCR was performed with the SYBR® Premix Ex Taq™ II kit (TAKARA) to identify gene expression. Relative expression levels of target genes were calculated by calibrating to the house-keeping gene β-actin as 2-(target gene Ct-reference gene Ct). All of the RT-PCR primer sequences are shown in Table2.

**Table 2:** The RT-PCR primer sequences in this study

Species	Target gene symbol	Sequence (5′–3′)
Rat	UBR1	F-CTTAGCGTTCCCGTCCTTGT
		R-GCCATGGTGACCAGATGGAA
	UBR2	F-TACCAACCAACCTCATCCGC
		R-AGTTTGTTGGCTCCTCTCGG
	UBR3	F-AGGCATGCAGAACAAGGGAA
		R-GGAACCTTGGTGCAGACACT
	UBR4	F-AGTGCAATGGACTCCTTCCG
		R-GCGCAGGAAAAGCAGTTTGA
	UBR5	F-CTGTCGGCAAGGTGTGCTTA
		R-GCTCTCTGGAGACCGAAGTT
	UBR6	F-CCCACAGTGGTTCGATGTGA
		R-ATCCATACGCCTGCGAAGTT
	UBR7	F-GCCACCTATTGGCCCTTGAA
		R-TGTCAGTTGCCTGGTCACTC
	β-actin	F-CTGGAACGGTGAAGGTGACA
		R-AAGGGACTTCCTGTAACAATGCA

F: forward; R: reverse.

### Western blot analysis

The cells were lysed with radioimmunoprecipitation assay (RIPA) lysis buffer [150 mM NaCl, 50 mM Tris–HCl (pH 7.4), 1% sodium deoxycholate, 1% NP-40, 1 mM PMSF and 1 mM ethylenediaminetetraacetic acid] at 4°C for 20 min. After centrifugation at 20,000 × g and 4°C for 10 min., 4× SDS gel sample buffer (Invitrogen) was added to the cleared lysate. The proteins were fractionated based on their molecular weight by SDS-PAGE (Invitrogen), transferred onto a polyvinylidene fluoride membrane (Invitrogen) at a constant current of 350 mA for 90 min. at 4°C and immunoblotted using the corresponding antibodies (anti-UBR3 and anti-UBR6 antibodies were obtained from Santa Cruz Biotechnology (Santa Cruz, CA, USA); anti-Na_v_1.5 antibodies were purchased from Sigma-Aldrich, St. Louis, MO, USA; anti-glyceraldehyde-3-phosphate dehydrogenase (GAPDH) antibodies were obtained from Cell Signaling (Danvers, MA, USA); anti-Ubiquitin antibodies were obtained from Abcam (Cambridge, MA, USA); horseradish peroxidase-conjugated secondary antibodies were obtained from Santa Cruz Biotechnology).

### Determination of Na_v_1.5 protein ubiquitination

Total proteins were extracted with RIPA buffer from HEK293 cells transfected with Na_v_1.5 plasmids, either alone or combined with UBR3/6 siRNA. They were incubated for 12 hrs by rotation at 4°C with either anti-Na_v_1.5 antibodies or the isotype control antibodies, added with protein-A/G-Sepharose beads (Beyotime, Shanghai, China), and incubated for a further 3 hrs to precipitate the protein-antibody complexes. Then, the precipitates were electrophoresed on a SDS gel, and immunoblotted with anti-Na_v_1.5 and anti-ubiquitin antibodies.

### Cycloheximide blocking assay

Cycloheximide (CHX), a specific inhibitor of protein synthesis that works by preventing the translocation of ribosomes, can effectively inhibit *de novo* protein synthesis in eukaryotic cells 20,21. This process was accomplished by treating UBR3/6 knockdown cells with or without CHX to test the additional translational inhibition. More specifically, NRVMs were transfected with the siRNA of UBR3/6 for 24 hrs. Next, we added 100 μg/ml CHX (Sigma-Aldrich). Aliquots of cells were collected at the 24-hr time-point and then subsequently at 4, 8 and 12 hrs after CHX addition. Protein was then extracted, and Western blot analysis was performed to analyse the levels of Na_v_1.5 channel proteins.

### Electrophysiological measurements

Standard voltage and current clamp techniques were used to assess the cardiac Na^+^ current and AP properties respectively 22,23. Whole-cell patch-clamp recordings were performed at room temperature (24°C) using an EPC-10 amplifier and pulse software (HEKA, Ludwigshafen, Germany) on the 2nd or 3rd day. Single cell cardiac electrophysiological properties were acquired from healthy NRVM. The extracellular solution (pH 7.4, titrated with NaOH) consisted of the following (in mM): NaCl 140, CsCl 10, CaCl_2_ 2, MgCl 21, glucose 5 and 4-(2-Hydroxyethyl)-1-piperazineethanesulfonic acid (HEPES) 10. The intracellular solution (pH 7.2, titrated with CsOH) contained the following (in mM): CsF 110, CsCl 10, NaF 10, ethylene glycol tetraacetate (EGTA) 11, CaCl_2_ 1, MgCl 21, Na_2_ATP 2 and HEPES 10.

### Statistical analysis

All of the data are presented as the mean ± SEM. Statistical differences among multiple groups were compared by one-way anova followed by the Fisher’s least significant difference test, using SPSS 13.0 (SPSS Inc., Chicago, IL, USA). *P* < 0.05 was considered statistically significant. Voltage-clamp data were compiled and analysed using Pulsefit (HEKA) and Origin 7.5 (OriginLab, Northampton, MA, USA). Single cell current amplitudes were normalized for differences in cell size by whole-cell membrane capacitance. Data were collected from at least three independent batches of experiments.

## Results

### Knockdown of UBR 3 and 6 elevates Na_v_1.5 channel protein expression

To analyse the potential roles of UBR1–7 in Na_v_1.5 expression, we first performed RT-PCR to test the mRNA expression of UBR1–UBR7 in rat cardiomyocytes. As shown in Figure1, all of the UBR members were expressed. UBR6 displayed the highest expression level, while UBR5 and UBR7 had the lowest expression. Next, using the gene silencing approach, we aimed to determine whether UBRs affected the protein expression of intracellular Na_v_1.5 channels. Considering the sequence similarity of UBR genes, we examined the specificity and efficiency of siRNA knockdown in NRVMs. After 48 hrs of transfection, the gene expression of the UBR family was tested by RT-PCR, and the results showed that UBR1–UBR7 siRNAs specifically interfered with their respective UBRs (Table3). Then, we measured the protein expression of Na_v_1.5 channels in UBR-deficient NRVMs. The Western blot data demonstrated that knockdown of UBR3 and UBR6 but not UBR1, UBR2, UBR4, UBR5 or UBR7 significantly increased the protein levels of intracellular Na_v_1.5 channels (Fig.2A and B). In another set of experiments with HEK293T cells expressing Na_v_1.5 channels, down-regulation of UBR3/6 showed effects on Na_v_1.5 that were similar to those observed in NRVMs (Fig.2C). These findings suggest that both UBR3 and UBR6 may play an important role in the regulation of intracellular Na_v_1.5 channel expression. Next, we examined the effects of UBR3–UBR6 double knockdown. The increase in Na_v_1.5 channel protein was also observed for UBR3–UBR6 double knockdown, which was comparable to that for the individual knockdown of either UBR3 or UBR6 (Fig.2D).

**Figure 1:** Quantitative PCR analysis of UBRs in NRVMs. The mRNA expression of every member of the UBR family could be detected in NRVMs. UBR2, UBR3, UBR4 and UBR6 had a relatively higher expression, while UBR5 and UBR7 were lower. All of the UBR1–7 primer pairs are listed in Table2. GAPDH served as a control (*n* = 3).

**Table 3:** The specificity and the efficiency of siRNA knockdown of UBR members

	UBR1	UBR2	UBR3	UBR4	UBR5	UBR6	UBR7
SiRNA of UBR1	++++	−	+	−	−	−	−
SiRNA of UBR2	−	++++	+	+	−	−	−
SiRNA of UBR3	+	+	+++	−	+	−	−
SiRNA of UBR4	−	−	−	++	−	−	−
SiRNA of UBR5	−	−	−	−	++++	−	−
SiRNA of UBR6	+	−	+	+	−	++++	+
SiRNA of UBR7	+	+	+	+	+	−	++++

++++ means the knockdown efficiency (decrease in protein level) >70%, +++ means 50–70%, ++ means 35–50%, + means 35–25%, − means <25%.

**Figure 2:** Protein expression of Na_v_1.5 channels in UBR knockdown cells. (A) *Left*. A typical example of a Western blot is shown using anti-Na_v_1.5 antibodies to assess the expression of Na_v_1.5 channel protein in NRVMs receiving different UBR siRNAs. Only UBR3/6 knockdown significantly changed Na_v_1.5 channel expression. GAPDH served as a loading control. *Right*. The pooled and quantified Western blot data. (B) Western blot analysis of Na_v_1.5 channels in UBR3/6 knockdown NRVMs. UBR3/6 significantly increased Na_v_1.5 expression in NRVMs. *Upper*. Western blot analysis and pooled data for Na_v_1.5 channels and UBR3 protein expression with or without transfection of UBR3 siRNA. GAPDH served as a loading control. *Lower*. Western blot analysis and pooled data using anti-Na_v_1.5 and anti-UBR6 antibodies to analyse Na_v_1.5 channel expression with or without transfection of UBR6 siRNA. GAPDH served as a loading control. (C) Western blot analysis in HNK293T cells expressing Na_v_1.5 channels after UBR3/6 knockdown. UBR3/6 could significantly increase Na_v_1.5 expression. *Upper*. Western blot and pooled data for Na_v_1.5 channels and UBR3 proteins level in HNK293T cells expressing Na_v_1.5 channels with or without UBR3 siRNA. GAPDH served as a loading control. *Lower*. Western blot analysis and pooled data using anti-Na_v_1.5 and anti-UBR6 antibodies to analyse Na_v_1.5 channel expression in HNK293T cells expressing Na_v_1.5 channels with or without UBR6 siRNA. GAPDH served as a loading control. (D) Western blot analysis of Na_v_1.5 channels in NRVMs. Cell were transfected with UBR3 and UBR 6 siRNA either alone or combined together. The scramble control RNA served as the control. *Left*. A typical example of a Western blot image for Na_v_1.5 channels and UBR3/6 protein expression. GAPDH served as a loading control. *Right*. Quantitative data for Western blots. All the data are from three independent experiments, *P < 0.01.

### UBR3/6 regulate the protein expression of Na_v_1.5 channels *via* degradation

The orchestration of mRNA transcription, protein translation, post-translational modification and protein degradation determines protein levels in cells. To understand the potential reasons underlying the increased Na_v_1.5 channel expression in UBR3/6-deficient cells, we first measured the mRNA expression of Na_v_1.5 channels. The RT-PCR results showed that UBR3/6 knockdown did not significantly change the mRNA level of Na_v_1.5 (Fig.3A). Next, CHX, an effective inhibitor of protein synthesis, was used to explore whether enhanced Na_v_1.5 protein synthesis contributed to its elevation in response to reduced levels of UBR3/6. Western blot data revealed that CHX treatment resulted in a time-dependent decrease in endogenous Na_v_1.5 levels in normal cells. Conversely, the pharmacological treatment did not counteract the increase in Na_v_1.5 protein caused by UBR3/6 knockdown (Fig.3B and C). Then, a proteasome activator SDS (0.003%) and a proteasome inhibitor MG132 (2 μM) were used to examine whether the proteasome pathway is involved in Na_v_1.5 protein degradation. As shown in Figure3D, SDS reduced Na_v_1.5 proteins, whereas MG132 increased Na_v_1.5 proteins. The additional application of UBR3/6 knockdown did not modify the increase in Na_v_1.5 proteins caused by MG132. These results suggest that UBR3 and UBR6 may degrade Na_v_1.5 channels through the proteasome way. To test whether ubiquitination mediated Na_v_1.5 degradation through proteasomes, we examined Na_v_1.5 ubiquitylation by immunoprecipitating Na_v_1.5 proteins followed by anti-ubiquitin immunoblotting, using HEK293T cells overexpressing Na_v_1.5. In Western blots for ubiquitylation, both unmodified Na_v_1.5 and ubiquitinated Na_v_1.5 were detected in the samples after immunoprecipitation (IP) with anti-Na_v_1.5 (Fig.3E). The ubiquitinated Na_v_1.5 displayed a larger molecular weight compared to the unmodified Na_v_1.5, and long-chain ubiquitylation of Na_v_1.5 is indicated by the molecular weight difference. In contrast to the very diffuse ubiquitylation band of whole-cell lysate (Fig.3E, upper panel, right lane), the bands of ubiquitinated Na_v_1.5 are concentrated (Fig.3E, upper panel, left 3 lanes), indicating that Na_v_1.5 proteins carry homogenous amounts of ubiquitin moieties. The amount of ubiquitinated Na_v_1.5 was remarkably reduced by the knockdown of either UBR3 or UBR6. The results showed that UBR3/6 knockdown reduced Na_v_1.5 ubiquitylation level, suggesting the stimulative effects of UBR3/6 on Na_v_1.5 ubiquitylation (Fig.3E).

**Figure 3:** *De novo* synthesis inhibiting assay and proteasome inhibiting assay of UBR3/6 knockdown-induced increases in Na_v_1.5 channels. (A) mRNA expression of Na_v_1.5 channels after UBR3/6 knockdown in NRVMs. UBR3/6 did not affect the mRNA level of Na_v_1.5 channels. *Left*. The efficiency of UBR3/6-siRNA knockdown in NRVMs. *Right*. The mRNA expression of Na_v_1.5 channels in UBR3/6 knockdown NRVMs. β-actin served as a control. (B) Effect of cycloheximide, an inhibitor for protein synthesis, on Na_v_1.5 channel expression in UBR3 knockdown NRVMs. NRVMs were transfected with or without UBR3 siRNA for 24 hrs prior to subsequent addition with cycloheximide (CHX) (100 μg/ml). Aliquots of the cells were collected at 4, 8 and 12 hrs after CHX treatment for Western blot analysis. A typical example of a Western blot analysis (left panel) and the summarized data (right panel) are shown (*n* = 3, *P < 0.01). Following CHX treatment, the endogenous Na_v_1.5 protein level showed a time-dependent decrease in cells receiving scramble control RNA. The increase in Na_v_1.5 protein in UBR3 knockdown cells was not counteracted. (C) Effect of cycloheximide on Na_v_1.5 channel expression in UBR6 knockdown NRVMs. NRVMs were transfected with or without UBR6 siRNA for 24 hrs prior to subsequent treatment with cycloheximide (CHX) (100 μg/ml). Aliquots of the cells were collected at 4, 8 and 12 hrs after CHX treatment for Western blot analysis. A typical example of a Western blot analysis (left panel) and the summarized data (right panel) are provided (*n* = 3, *P < 0.01). Following CHX treatment, the endogenous Na_v_1.5 protein level showed a time-dependent decrease in scramble control cells. The UBR3/6 reduction-induced increase in Na_v_1.5 protein was not counteracted. (D) Effect of proteasome activation and inhibition on Na_v_1.5 protein levels in NRVMs. SDS (0.003%) and MG132 (2 μM) were used to activate and inhibit proteasomes respectively. SDS was incubated for 24 hrs before the harvest of NRVMs. Individual or combined siRNAs against UBR3 and UBR6 were transfected for 12 hrs prior to subsequent addition with MG132 for a further 24 hrs. A typical example of a Western blot analysis (left panel) and the summarized data (right panel) are provided (*n* = 3, *P < 0.01). (E) Examination of Na_v_1.5 protein ubiquitination in Na_v_1.5-overexpressing HEK293 cells receiving UBR3/6 knockdown. Cell lysates were immunoprecipitated with anti-Na_v_1.5 antibodies (IP: Na_v_1.5), then immunoblotted with anti-ubiquitin (IB: Ub-Na_v_1.5) and anti-Na_v_1.5 (IB: Na_v_1.5) antibodies. *Position of unmodified Na_v_1.5. The image is a representative from three independent experiments.

### Reduced levels of UBR3/6 enhance the opening of Na_v_1.5 channel and thereby the amplitude of the action potential

Given the putative roles of Na_v_1.5 in the generation of an AP and the effects of UBR3/6 on Na_v_1.5 expression, we further measured Na^+^ currents and APs in NRVMs with or without UBR3/6 siRNA (Fig.4). We found that knockdown of UBR3/6 did not change the shape of the I–V curve of the Na_v_1.5 channel but significantly increased the peak current density (*P* < 0.01) (Fig.4A and B). The peak current density generated by the Na_v_1.5 channels in UBR3 knockdown cells increased from (−51.49 ± 7.735) pA/pF to (−75.94 ± 13.43) pA/pF (*n* > 10; *P* < 0.01). The peak current density of the Na_v_1.5 channels in UBR6 knockdown cells could be elevated from (−51.49 ± 7.735) pA/pF to (−87.06 ± 10.22) pA/pF (*n* > 10; *P* < 0.01). However, there was no change in the activation curve in UBR3/6-deficient and normal cells (Fig.4C). Moreover, both UBR3 and UBR6 knockdown significantly increased the amplitude of the AP (Fig.4D and E). These results suggest that UBR3/6 regulate Na_v_1.5 channel opening and AP in cardiomyocytes.

**Figure 4:** Effects of UBR3/6 knockdown on Na_v_1.5 channel currents and action potentials. (A) Representative tracings of Na_v1.5_ currents from rat cardiomyocytes. The amplitude of the UBR3/6 knockdown cells was increased. (B) Current–voltage (I–V) relationship of transient I_N__a_ from rat cardiomyocytes (*n* > 10 per group *P < 0.01). The current traces were recorded at V_m_ in the range of −70 to +40 mV from a holding potential of −120 mV. The I_N__a_ density of the UBR3/6 knockdown cells was elevated compared to the NC. (C) The activation curve for Na_v_1.5 channels from NC (negative control) and UBR3/6 knockdown rat cardiomyocytes (*n* > 10 per group). There were no significant differences between them. (D) Representative AP (action potential) recordings from NC (negative control) and UBR3/6 knockdown rat cardiomyocytes. (E) Statistical analysis of the amplitude of the APA (action potential amplitude) (*n* > 10 per group, *P < 0.01). The amplitude was increased in UBR3/6 knockdown cells.

## Discussion

In the present study, we investigated the effects of UBR isoforms on the expression of cardiac Na_v_1.5 channels. We found that only UBR3 and UBR6 affected the protein levels of Na_v_1.5 channels. The UBR3/6-mediated regulation of Na_v_1.5 channels was not transcriptionally mediated but was associated with the ubiquitin–proteasome degradation system. Furthermore, UBR3/6 knockdown enhanced the opening of Na_v_1.5 channels and thereby the amplitude of APs. Overall, we identified a new regulatory function of UBR3 and UBR6 in cardiac electrophysiology by the degradation of Na_v_1.5 protein.

Ubiquitination is a key step in the ubiquitin–proteasome pathway, which serves as an important regulator for plasma membrane proteins in their trafficking, internalization and degradation 24. Once ubiquitylated, the internalized membrane proteins can be targeted for lysosomal or proteasomal degradation 8. In the UPS, E3 ligase is the key enzyme in recognizing the specificity degradation signals of substrate ubiquitylation 11. UBR box family is a unique class of E3 ligase that recognize N-degrons or structurally related determinants for ubiquitin-dependent proteolysis and perhaps other processes as well. The mammalian genome encodes at least seven UBR box-containing proteins, called UBR1 to UBR7 25. UBR1 is a 225-kD RING-type E3 ligase containing at least three substrate-binding sites 25. The mouse UBR1 and UBR2 are 200-kD N-recognins with 47% identity and 68% similarity to each other, and are functionally overlapped 26. UBR3 is a 213-kD RING finger E3, shares weak but detectable homology to UBR1 and UBR2 25. UBR4 is an exceptionally large protein with a MW of 570-kD, and UBR5 (300-kD) is also known as EDD/Hhyd. Phylogenetic analysis of the UBR box motif sequences from yeast to mouse classified them into the following subfamilies: UBR1/2/3 (with the RING finger), UBR4, UBR6 (with an F-box), UBR5 (with the HECT domain) and UBR7 (with the plant homeodomain) 25. In recent studies, Na_v_1.5 has been reported to be internalized by the ubiquitin E3 ligase Nedd4-2, and thus down-regulated from its functional expression 27,28. However, the internalization of Na_v_1.5 by Nedd4-2 does not seem to be linked to degradation as there was no reduction in the total level of Na_v_1.5 protein upon co-expression with Nedd4-2 1,8,10. In contrast, another study found that pharmacological inhibition of the proteasome was linked to an increase in Na_v_1.5 expression and I_Na_ in neonatal rat cardiomyocytes 5. However, it is unclear whether any ubiquitin E3 ligases target Na_v_1.5 for the ubiquitin–proteasome degradation pathway. The UBR family has been described to be involved in the function of olfactory and other sensory systems 14, neurogenesis and cardiovascular development 15, and genome stability 17,29. Nevertheless, the roles of UBR family members in cardiomyocytes remain unknown. In the present study, we sought to elucidate the relationships between UBRs and Na_v_1.5 expression. Our results showed that individual knockdown of UBR3 and UBR6, but not other UBR isoforms, increased the protein levels of Na_v_1.5 channels in neonatal rat cardiomyocytes. Next, we confirmed that this regulation of Na_v_1.5 channels by UBR3/6 was not transcriptionally mediated as the inhibition of *de novo* protein synthesis did not affect the increase in Na_v_1.5 proteins upon UBR3/6 knockdown. We further observed that the inhibition of proteasomes with MG132 abolished the effects of UBR3/6 knockdown (Fig.3D), and that UBR3/6 knockdown reduced Na_v_1.5 ubiquitylation (Fig.3E). These results strongly suggest that UBR3/6 promote Na_v_1.5 ubiquitylation and degradation through proteasomes. Interestingly, we observed complete stabilization of Na_v_1.5 proteins with single knockdown of either UBR3 or UBR6. Besides, double UBR3–UBR6 knockdown resulted in similar increases of Na_v_1.5 proteins, compared to those obtained with single knockdown (Figs2D and 3D). It is likely that UBR3 and UBR6 act in concert to promote degradation of Na_v_1.5. Another possibility is that UBR3 and UBR6 may take effect through similar mechanisms. The covalent binding sites on Na_v_1.5 for ubiquitylation are theoretically limited. UBR3 and UBR6 may induce the same ubiquitylation level at the same ubiquitylation sites. Thus, single or combined knockdown of UBR3 and UBR6 may take the same effect. Notably, unlike UBR1, UBR2 or UBR4, although UBR3 and UBR6 belong to the UBR family, they are not bound to the known N-end rule substrates 25,30. UBR3 and UBR6 may have other non-N-end rule physiological ligands. The details of UBR3 and UBR6 on Na_v_1.5 protein ubiquitylation remain to be elucidated. Despite that, our observations revealed the regulation of UBR3 and UBR6 on Na_v_1.5 protein levels through the ubiquitin–proteasome degradation pathway. To our knowledge, UBR3 and UBR6 are the first E3 members observed to be linked to the degradation of Na_v_1.5 through proteasomes.

To examine the interaction between UBR3/6 and Na_v_1.5, we performed co-IP to check whether Na_v_1.5 binds to UBR3/6, using HEK293T cells overexpressing Na_v_1.5 proteins. However, no significant binding was shown by the co-IP tests (data not shown). The reasons may lie in technical issues. The amount of Na_v_1.5 proteins expressed by HEK293T cells might be too small to be detected by co-IP, and the weak and transient interaction between UBR3/6 and Na_v_1.5 may not allow its detection by co-IP. Also, there is a possibility that the action of UBR3/6 on Na_v_1.5 ubiquitylation and degradation is not direct but occurs through other ligases, such as Nedd4-2 that has been described previously 1,10. More study is required to determine whether UBR3/6 directly take effect on Na_v_1.5 or not.

The major cardiac voltage-gated sodium channel Na_v_1.5 plays a key role in the generation of AP. The opening and closing of this channel can regulate the flow of Na^+^ and control the voltage gradient between the inside and outside of cells to initiate AP and conduct electrical impulses 31,32. Abnormalities of the Na_v_1.5 channel may distort AP and thereby lead to different types of arrhythmia syndromes and some congenital and acquired cardiac disorders 33–35. Based on the present evidence, the molecular mechanisms associated with Na_v_1.5 in these diseases are multitudinous. Na_v_1.5-associated proteins that can regulate its synthesis, transportation, structure, activity and degradation may also be associated with its function. In contrast to the numerous mutations found in the *SCN5A* gene 36, the number of related proteins that can regulate Na_v_1.5 expression is limited 9,37. Deletion of forkhead box protein O1 enhance the expression of cardiac Na_v_1.5, increase Na^+^ channel activity and result in a shortened QRS 38. In contrast, defects in the PDZ domain-binding motif of Na_v_1.5 may reduce its expression and the sodium current in the lateral myocyte membrane, leading to increased anisotropy of the ventricular conduction and Brugada syndrome 39. This finding suggests that Na_v_1.5 expression is a crucial step in its normal function in cardiomyocytes.

In the present study, we discovered two new regulators of Na_v_1.5 expression that could reduce the protein levels of Na_v_1.5 channels by ubiquitination. The UBR3/6-mediated degradation of Na_v_1.5 affected the opening of ion channels and thereby the amplitude of APs. This discovery has certain pathophysiological implications, suggesting a potential association of UBR3/6 with heart diseases such as arrhythmias. UBR3 and UBR6 might serve as potential targets for therapeutic intervention in ion channel diseases.
